The article "Loss of FOXN3 in colon cancer activates beta-catenin/TCF signaling and promotes the growth and migration of cancer cells" was retracted in 2026. Reasons: results that could not be reproduced; errors in the materials; plagiarized images; duplicated images.

# Loss of FOXN3 in colon cancer activates beta-catenin/TCF signaling and promotes the growth and migration of cancer cells

**DOI:** 10.18632/oncotarget.14189

**Published:** 2016-12-26

**Authors:** Yuedi Dai, Meixing Wang, Haixia Wu, Mi Xiao, Houbao Liu, Dexiang Zhang

**Affiliations:** ^1^ Department of Medical Oncology, Cancer Hospital of Fudan University, Minhang Branch, Shanghai 200240, China; ^2^ General Surgery Department, General Surgery Institute, Zhongshan Hospital, Fudan University, Shanghai 200032, China; ^3^ General Surgery Department, The Fifth People's Hospital of Shanghai, Fudan University, Shanghai 200240, China

**Keywords:** FOXN3, colon cancer, beta-catenin/TCF signaling, cell growth and migration

## Abstract

Aberrant activation of beta-catenin/TCF is a hallmark of colon cancer. How the functions of nuclear localized beta-catenin are regulated is not fully understood. Here, it was found that FOXN3 (Forkhead box N3) was down-regulated in colon cancer tissues. Forced expression of FOXN3 inhibited the growth, migration and invasion of colon cancer cells, while knocking down the expression of FOXN3 promoted the growth, migration, invasion and metastasis of colon cancer cells. FOXN3 bind to beta-catenin and inhibited beta-catenin/TCF signaling by blocking the interaction between beta-catenin and TCF4. Taken together, these data demonstrated the suppressive roles of FOXN3 in the progression of colon cancer, and indicated that restoring the functions of FOXN3 would be a novel therapeutic strategy for colon cancer.

## INTRODUCTION

Colon cancer is one of the most common malignancies in the world [1, 2]. Activation of wnt/beta-catenin signaling is one of the hallmarks of this malignancy [3]. Although multiple genetic mutations have been found to activate wnt/beta-catenin signaling and lead to the nuclear accumulation of beta-catenin [4–6], the regulation of nuclear beta-catenin was not fully understood.

Wnt/beta-catenin signaling has been demonstrated to promote the progression of colon cancer [7]. In the absence of Wnt ligand, Axin, APC, CK1 and GSK3 beta form a destruction complex, which promotes the phosphorylation of beta-catenin at its N-terminal Ser/Thr residues by CK1 and GSK3 beta. The phosphorylated beta-catenin is ubiquitinated and undergoes degradation. Upon the stimulation of wnt ligand, the formation of destruction complex is inhibited, which resulted in the β-catenin stabilization and translocation into nucleus. In the nucleus, beta-catenin binds with transcription factors of the TCF/LEF-1 family, leading to the increased expression of oncogenic genes, such as c-Myc and cyclin D1 and Snail [8, 9]. Aberrant activation of wnt/beta-catenin signaling promotes the growth, migration and metastasis of colon cancer cells [10, 11]. Therefore, targeting the Wnt/beta-catenin signaling pathway is a promising strategy for the treatment of colon cancer.

FOXN3 (also named CHES1) was first identified in the yeast as a suppressor of check point defects [7]. Like other members of forkhead transcriptional factors, FOXN3 bind with a panel of nuclear proteins, such as MEN1, HDAC1, HDAC2, and so on [7]. Several studies have reported the physiological functions of FOXN3 in the embryonic development [12, 13]. Recently, down-regulation of FOXN3 has been observed in several cancer types, including hepatocellular carcinoma, oral squamous cell carcinoma, laryngeal cancer and diffuse large B-cell lymphoma [14–16]. However, the molecular mechanisms through which down-regulation of FOXN3 promoted the tumorigenesis remain poorly understood.

In this study, we have examined the expression of FOXN3 in the colon cancer tissues, studied the functions of FOXN3 in the progression of colon cancer and investigated the molecular mechanisms.

## RESULTS

### The expression of FOXN3 was down-regulated in colon cancer

To study the expression pattern of FOXN3 in colon cancer, we first turned to a dataset available in the Oncomine database. According to the gene expression profile, in the sample considered (composed of 19 normal colon tissues, 3 normal rectum tissues and 101 colon adenocarcinoma tissues), the expression was lower in colon adenocarcinoma tissues when compared with the normal colon tissues. The median log2 expression value of FOXN3 decreases from about 1.3 of normal to -0.2 of colon adenocarcinoma (Figure 1A). To confirm the results from the analysis of dataset available in the Oncomine database, we examined the mRNA level of FOXN3 in 30 colon cancer tissues and paired non-cancerous adjacent tissues. Consistent with the observations in Figure 1A, decreased FOXN3 mRNA level was found in colon cancer tissues (Figure 1B). Furthermore, the results from the immnohistochemistry and western blot analysis confirmed the down-regulation of FOXN3 protein in colon cancer tissues (Figure 1C–1D). In addition, the protein level of FOXN3 in a panel of normal colon epithelial cells and colon cancer cells was examined. Lower FOXN3 protein level in colon cancer cells (SW620, SW480 and HCT8) and higher FOXN3 protein level in normal colon epithelial cells (HIEC and NCM460) were observed (Figure 1E). Finally, we examined the expression of FOXN3 in the colon cancer mouse model driven by Ras^G12D^ and loss of P53 (Figure 1F). The expression of Villin-Cre induced the expression of Ras^G12D^ and knocking down the expression of P53, and ultimately led to the colon adenocarcinoma (Figure 1F). The expression of FOXN3 in normal colon tissues and tumors was examined by western blot analysis. The protein level of FOXN3 in the colon tissues from Villin-Cre; LSL-Ras^G12D^; P53^f/f^ was dramatically decreased (Figure 1G). Taken together, these data suggested that the expression of FOXN3 was decreased in colon cancer.

**Figure 1:** The expression of FOXN3 was decreased in colon cancer **A**. The results from Oncomine database showed the down-regulation of FOXN3 in colon adenocarcinoma. Boxplot of FOXN3 mRNA Log2 expression levels was evaluated in Oncomine database. This study contained 19 normal colon tissues, 3 normal rectum tissues and 101 colon adenocarcinoma tissues. **B**. The expression of FOXN3 mRNA was down-regulated in colon cancer tissues compared with the paired normal tissues. The FOXN3 mRNA level was examined in 30 colon cancer tissues and the paired normal tissues using Real-time PCR. The expression of FOXN3 mRNA level was normalized to 18S. **C**. The expression of FOXN3 protein in colon cancer tissues and paired non-cancerous tissues was examined using immunohistochemistry. **D**. The expression of FOXN3 protein in four colon cancer tissues and paired non-cancerous tissues was examined using western blot analysis. **E**. The expression of FOXN3 in normal colon cells and colon cancer cells. **F**. Tumors formed in colon cancer mouse model Villin-Cre; P53^f/f^; Ras^G12D^. **G**. The expression of FOXN3 protein was down-regulated in the colon tissues of the mouse Villin-Cre; P53^f/f^; Ras^G12D^.

### FOXN3 inhibited the growth and migration of colon cancer cells

To evaluate the roles of FOXN3 in the progression of colon cancer, we forced expression of FOXN3 in the SW480 and SW620 cells (Figure 2A). MTT assay, cell migration assay, soft agar assay and invasion assay were performed to examine the effects of FOXN3 on the growth, migration, anchorage-independent growth and invasion of colon cancer cells. It was found that over-expression of FOXN3 inhibited the growth of colon cancer cells (Figure 2B). Moreover, over-expression of FOXN3 inhibited the migration of colon cancer cells (Figure 2C). Furthermore, up-regulation of FOXN3 impaired the anchorage-independent growth of SW620 cells in the soft agar (Figure 2D). In addition, the increased expression of FOXN3 attenuated the invasion of colon cancer cells in the assay using transwells (Figure 2E). These data indicated the suppressive the roles of FOXN3 in the progression of colon cancer.

**Figure 2:** Forced expression of FOXN3 inhibited the growth, migration and invasion of colon cancer cells **A**. FOXN3 was over-expressed in SW480 and SW620 cells. **B**. FOXN3 inhibited the growth of SW480 and SW620 cells in the MTT assay. **C**. FOXN3 inhibited the migration of SW480 and SW620 cells in the Boyden chamber assay. **D**. FOXN3 inhibited the anchorage-independent growth of SW480 and SW620 cells in the soft agar assay. **E**. FOXN3 inhibited the invasion of SW480 and SW620 cells in the transwell assay.

To further clarify the functions of FOXN3 in the colon cancer, we knocked down the expression of FOXN3 in SW480 and SW620 cells (Figure 3A). Consistent with the results shown Figure 2B, knocking down the expression of FOXN3 promoted the growth of SW480 and SW620 cells in the MTT assay (Figure 3B). The cell cycle analysis showed that knocking down the expression of FOXN3 promoted the cell cycle progression (Figure 3C). Moreover, down-regulation of FOXN3 enhanced the migration of colon cancer cells in the assay using a modified Boyden chamber (Figure 3D). Furthermore, knocking down the expression of FOXN3 promoted the anchorage-independent growth of SW620 cells in the soft agar (Figure 3E). Additionally, down-regulation of FOXN3 facilitated the invasion of SW480 and SW620 cells (Figure 3F). Taken together, these data provided a good explanation for the down-regulation of FOXN3 in colon cancer.

**Figure 3:** Down-regulation of FOXN3 promoted the growth, migration and invasion of colon cancer cells **A**. FOXN3 was knocked down in SW480 and SW620 cells. **B**. Knocking down the expression of FOXN3 promoted the growth of SW480 and SW620 cells in the MTT assay. **C**. Knocking down the expression of FOXN3 promoted the Cell cycle progression. **D**. Knocking down the expression of FOXN3 promoted the migration of SW480 and SW620 cells in the Boyden chamber assay. **E**. Knocking down the expression of FOXN3 promoted the anchorage-independent growth of SW480 and SW620 cells in the soft agar assay. **F**. Knocking down the expression of FOXN3 promoted the invasion of SW480 and SW620 cells in the transwell assay.

### Knocking down the expression of FOXN3 activated beta-catenin/TCF signaling

To explore the potential mechanisms through which FOXN3 inhibited the growth, migration and invasion of the colon cancer cells, we examined the expression of FOXN3 on the activity of various signaling pathways using luciferase reporter assay. It was found that over-expression of FOXN3 inhibited the activity of Topflash, an indicator for beta-catenin/TCF signaling both at the basal level and upon the treatment of LiCl (Figure 4A). Moreover, knocking down the expression of FOXN3 up-regulated the expression of N-cadherin, Snail and c-Myc (three downstream genes downstream of beta-catenin/TCF signaling), indicating the activation of beta-catenin/TCF signaling (Figure 4B). ICG001 has been reported to block beta-catenin/TCF signaling. Here, it was found that ICG001 blocked the enhancement in the anchorage-independent growth, migration and invasion of colon cancer cells which was induced by knocking down the expression of FOXN3 (Figure 4C–4E). In summary, these data suggested that down-regulation of FOXN3 promoted the growth, migration and invasion of colon cancer cells by activating beta-catenin/TCF signaling.

**Figure 4:** Down-regulation of FOXN3 activated beta-catenin/TCF signaling in colon cancer cells **A**. Over-expression of FOXN3 inhibited the activity of Topflash, an indicator for beta-catenin/TCF signaling, both at the basal level and upon the stimulation of LiCl. **B**. Knocking down the expression of FOXN3 up-regulated the expression of N-cadherin, Snail and c-Myc. **C**. ICG001, the inhibitor for beta-catenin/TCF signaling, abolished the advantage on the anchorage-independent growth induced by knocking down the expression of FOXN3. **D**. ICG001abolished the advantage on the migration of SW620 cells induced by knocking down the expression of FOXN3. **E**. ICG001abolished the advantage on the invasion of SW620 and SW480 cells induced by down-regulation of FOXN3.

### FOXN3 inhibited the interaction between beta-catenin and TCF4

Since FOXN3 has been recognized as a transcriptional factor and belongs to the forkhead protein family, we first tested the interaction between beta-catenin and FOXN3. The fusion protein GST-FOXN3 pulled the beta-catenin down from the SW620 cell lysates, indicating the interaction between FOXN3 and beta-catenin (Figure 5A). In addition, over-expression of beta-catenin (Flag-beta-catenin) and FOXN3 (myc-FOXN3) in SW620 cells revealed the interaction between beta-catenin and FOXN3 in the immunoprecipitation assay (Figure 5B). Moreover, immunoprecipitation assay showed that the endogenously expressed beta-catenin and FOXN3 formed a complex in SW620 and SW480 cells (Figure 5C). Furthermore, we have found that exogenously expressed FOXN3, TCF4 and beta-catenin formed a complex in 293T cells using the sequential immunoprecipitation (Figure 5D). These observations confirmed the interaction between beta-catenin and FOXN3. In the nucleus, TCF4 has been reported to bind with beta-catenin and initiated the transcription. Therefore, we next examined whether FOXN3 inhibited the interaction between beta-catenin and TCF4. As shown in Figure 5E, forced expression of FOXN3 (myc-FOXN3) impaired the interaction between beta-catenin (Flag-beta-catenin) and TCF4 (HA-TCF4). These data demonstrated that FOXN3 inhibited beta-catenin/TCF signaling by blocking the interaction between TCF4 and beta-catenin.

**Figure 5:** FOXN3 bind with beta-catenin and blocked the interaction between beta-catenin and TCF in colon cancer cells **A**. The interaction between GST-FOXN3 and beta-catenin was demonstrated in the GST pull-down assay. **B**. Exogenously expressed beta-catenin (Flag-beta-catenin) and FOXN3 (myc-FOXN3) formed a complex in SW620 cells in the immunoprecipitation assay. **C**. Endogenously expressed beta-catenin and FOXN3 formed a complex in SW620 and SW480 cells. **D**. The sequential immunoprecipitation assay demonstrated that FOXN3 formed a complex with beta-catenin and TCF4 in293T cells. **E**. The immunoprecipitation assay demonstrated that FOXN3 inhibited the interaction between beta-catenin and TCF4.

### Knocking down the expression of FOXN3 promoted the metastasis of colon cancer cells

The observations that down-regulation of FOXN3 promoted the migration of colon cancer cells prompted us to examine whether knocking down the expression of FOXN3 promoted the metastasis of colon cancer cells *in vivo*. SW480 cells were labeled with a luciferase expression vector (SW480-Luci), which enabled the tracing of SW480 cells *in vivo* by an *in vivo* imaging system after administration of luciferin (the substrate of luciferase). The SW480-Luci cells were knocked down the expression of FOXN3 and injected into the nude mice through left ventricle. The metastasis of SW480-Luci cells was monitored by the *in vivo* imaging system. Knocking down the expression of FOXN3 enhanced the metastasis of SW480 cells which was demonstrated by the higher intensity of fluorescence from the mice injected with FOXN3 knocking down cells (Figure 6A–6B). To further examine the functions of FOXN3 in the metastasis of colon cancer cells, we examined the metastasis foci in colon. Knocking down the expression of FOXN3 promoted the tumorigenesis of colon cancer cells in the colon tissues (Figure 6C–6D). In summary, these results suggested that down-regulation of FOXN3 promoted the metastasis of colon cancer cells.

**Figure 6:** Knocking down the expression of FOXN3 promoted the metastasis of colon cancer cells **A-B**. Knocking down the expression of FOXN3 promoted the metastasis of SW480 cells. Cells were injected into the nude mice through the left ventricle of the heart. The intensity of the fluorescence was quantified. **C-D**. Knocking down the expression of FOXN3 promoted the distant seeding and metastaic foci formation of SW480 cells in the colon tissues. Classic hematoxylin and eosin staining of the colon tissues was performed and the metastatic foci were quantified.

## DISCUSSION

Up to date, the biological functions of FOXN3 remain poorly understood. Several studies have demonstrated the physiological functions of FOXN3 in the eye development of xenopus laevis and craniofacial development of mouse [12, 13]. In the pathological context, down-regulation has been observed in HCC and other cancer types [14], while the underlying mechanisms remain largely unknown.

In this study, we explored the expression pattern of FOXN3 in colon cancer. Down-regulation of FOXN3 in the colon cancer was observed both at the protein level and mRNA level, suggesting that the expression of FOXN3 might be a diagnosis marker for the colon cancer. Although we did not examine the mechanisms for the down-regulation of FOXN3 in colon cancer, several previous studies have provided some hints. For example, it has been reported that miR-574-5p down-regulated the expression of FOXN3 in lung cancer and promoted the progression of the tumor, suggesting the regulation of FOXN3 by microRNAs.

In the functional study, FOXN3 was found to suppress the growth, migration, invasion and colony formation of the colon cancer cells. Consistent with our observations, Sun et al have reported that FOXN3 inhibited the proliferation of HCC cells [14]. These studies further emphasized the suppressive effects of FOXN3 on the proliferation of cancer cells.

Although several studies have shown that FOXN3 expression is lost in the malignancies, much less is known concerning the underlying mechanisms. In this study, we have examined the effects of FOXN3 on the activity of several pathways. It was found that FOXN3 inhibited the activity of beta-catenin/TCF complex, which was demonstrated by the reporter assay and the expression of its downstream genes. It seemed that FOXN3 inhibited the interaction between beta-catenin and TCF4. These observations provided a good explanation for the suppressive roles of FOXN3 in colon cancer. Also, in our study, knocking down the expression of FOXN3 promoted the growth, migration, colony formation and invasion of colon cancer cells, which was abolished by ICG001, the inhibitor of beta-catenin/TCF signaling. The rescue effects of ICG001 further confirmed the activation of beta-catenin/TCF signaling upon knocking down the expression of FOXN3.

In summary, this study revealed the suppressive roles of FOXN3 in the progression of colon cancer. Further study using FOXN3 knock out mice would provide novel insights into its functions.

## MATERIALS AND METHODS

### Clinical colon cancer tissues

30 clinical colon cancer tissues and paired non-cancerous adjacent tissues were collected from patients who received surgery at Cancer Hospital of Fudan University, Fudan University. All of the patients agree with this study. This study was approved by the ethics committee of the hospital. Tissues were stored at -80°C in a freezer.

### Cell culture

Colon cancer cell lines (SW480, SW620 and HCT8) and normal human colon epithelial cell line (HIEC and NCM460) were obtained from ATCC (American Typical Culture Center). All cells were cultured in DMEM medium supplemented with 10% fetal bovine serum (GIBCO), 100units/mL penicillin and 100μg/mL streptomycin in an incubator with 5% CO_2_ at 37°C.

### Q-PCR analysis

TRIzol was used to exact total RNA. The complementary DNA (cDNA) was prepared using the reverse transcription kit. The expression of FOXN3 in the colon cancer tissues and paired normal tissues was examined by quantitative real-time PCR using SYBR® Green Realtime PCR Master Mix (TOYOBO) following the instructions of the manufacturer. Sequences of quantitative real-time PCR primers are listed as follows:

18S Forward primer: 5′-TAAATCAGTT ATGGTTCCTT -3′

18S Reverse primer: 5′-CGACTACCATCGAA AGTTGA-3′

FOXN3 Forward primer: 5′-GAATTAGTGTCTCC AGTGGA-3′

FOXN3 Reverse primer: 5′-TCTTCAGCAAGTT CTTGCTC-3′

### Immunohistochemistry

Formalin-fixed, paraffin-embedded tissue sections (5μm) were deparaffinized in xylene and rehydrated with gradient concentrations of ethanol. Endogenous peroxidase activity was blocked (0.35% H2O2 in PBS buffer), antigens were retrieved by microwaving (350 W), and nonspecific binding was blocked by 1% bovine serum albumin in PBS buffer. Sections were incubated with FOXN3 antibody (1:300) over night. After extensive wash with PBS, the sections were incubated with the HRP-linked secondary antibody (Envision, DakoCytomation) for 1 hour. Slides were then incubated with 3, 3′-diaminobenzidine chromogen (DakoCytomation), counterstained in Meyer's hematoxylin and mounted.

### Western blot

Whole cell lysates were prepared using RIPA buffer. The cellular proteins were resolved by SDS-PAGE. Then the proteins were transferred to the PDVF membrane. After blocking with 3% BSA, the membrane was incubated with following primary antibodies over night: anti-FOXN3 (Abcam, 1:2000), anti-Snail (Cell Signaling Technology, 1:1000), anti-Cyclin D1 (Abcam, 1:1000), anti-c-Myc and anti-GAPDH (Santa Cruz, 1:1000). The membranes were washed with TBST solution and incubated with the secondary antibody for 1 hour at the room temperature. The protein was visualized by ECL kit.

### GST pull-down assay

The coding sequence of FOXN3 was inserted into the expression vector pGEX-4T-1. The fusion protein GST-FOXN3 was purified. The whole cell lysates of SW620 were prepared in 50 mM Tris-Cl (pH 7.5), 150 mM NaCl, 0.1% NP40 and protease inhibitor cocktail. 5 μg GST-FOXN3 fusion protein and 800 μg cell lysates were incubated at 4°C for 3 hr. 20 μl of glutathione-Sepharose-4B beads were added to the samples and incubated at 4°C for 1 hr to capture the GST fusion proteins. After washing with lysis buffer three times, the proteins were eluted in Laemmli buffer and analyzed by SDS-PAGE.

### Luciferase assay

SW620 Cells were plated at a subconfluent density. 18 hours later, the reporter assays were performed using 0.1 μg of Topflash, 0.5 μg of expression vector, and 0.05 μg of TK Renilla luciferase (internal control for transfection efficiency). 48 hours later, cells were treated with 25mM LiCl or NaCl for 8 hours. Then, cell lysates were prepared and the reporter activity was measured using the dual-luciferase reporter assay system (Promega).

### Construction of vectors

The coding sequence of FOXN3 was amplified by PCR and inserted into the expression vector pcDNA3.1 to obtain the myc tagged FOXN3. The coding sequence of beta-catenin was amplified by PCR and inserted into the expression vector pCMVTag2B to obtain the Flag tagged beta-catenin. The coding sequence of TCF4 was amplified by PCR and inserted into the expression vector pCMV-HA to obtain the HA tagged TCF4.

### Knocking down the expression of FOXN3

RNAi lenti-virus particles (sicon and siFOXN3) were purchased from GeneChem (China). Cells were infected with the indicated lenti-virus particles of the same MOI for 24 hours and then stable knock-down cells were selected with the medium containing puromycin for at least a week.

### MTT assay

Cells were plates in 96-well plates at the density of 10^5^ cells/well. Cell growth was determined using the 3-(4,5-methylthiazol-2-yl)-2,5-diphenyltetrazolium bromide (MTT) colorimetric growth assay for a week. Every other day, cell growth was determined by adding MTT solution (50μg/well) for 4h. Cellular MTT was resolved with DMSO and was measured at 540 nm. All experiments were performed in triplicates.

### Boyden chamber assay

Cell migration was examined using Boyden chamber. Cells (2×10^5^) suspended in 0.05ml medium containing 1% FBS were placed in the upper chamber, and the lower chamber was loaded with 0.152ml medium containing 10% FBS acting as the chemoattractant. 12 hours later, cells migrated to the lower surface of filters was detected with traditional hematoxylin and eosin (H&E) staining. The experiments were repeated for three times. Five random visual fields were counted for each sample and the average was determined.

### Mice model

Mice were housed and treated after being approved by the Institutional Animal Care and Use Committee of Fudan University. *Kras^G12D^;P53 ^f/f^* and *Villin-Cre* mice were obtained from Jacks Lab (Koch Institute for Integrative Cancer Research, Cambridge, MA). *Kras^G12D^* strain carries a point mutation (G12D) in the Kras (v-Ki-ras2 Kirsten rat sarcoma viral oncogene homolog) gene whose expression is blocked by the presence of a loxP-flanked stop codon. Cre-mediated recombination can excise the stop codon and permit the oncogenic protein to be expressed. Colon cancer mouse models *Villin-Cre; Kras^G12D^*; *P53 ^f/f^* and *Kras^G12D^*; *P53 ^f/f^* mice were generated by crossing *Kras^G12D^*; *P53 ^f/f^* and *Villin-Cre* mice.

### Statistical analysis

Statistical analyses were performed by the Student t-test (two-tailed) using Prism GraphPad software. Differences with *P* < 0.05 were considered statistically significant. Data were represented as mean±SEM.

## Abbreviations

TCF4: T-cell factor 4
ATCC: American Type Culture Collection
DMEM: Dulbecco's modified Eagle's medium
GFP: green fluorescence protein
FBS: fetal bovine serum
RT-PCR: Reverse transcription quantitive PCR
cDNA: Complementary DNA
PBS: phosphate-buffered saline.
